# MicroRNA-542-3p inhibits oral squamous cell carcinoma progression by inhibiting ILK/TGF-β1/Smad2/3 signaling

**DOI:** 10.18632/oncotarget.19986

**Published:** 2017-08-07

**Authors:** Bin Qiao, Jing-Hua Cai, Alfred King-Yin Lam, Bao-Xia He

**Affiliations:** ^1^ Department of Stomatology, The First Affiliated Hospital of Zhengzhou University, Zhengzhou 450052, P.R. China; ^2^ Cancer Molecular Pathology, School of Medicine and Menzies Health Institute Queensland, Griffith University, Gold Coast 4222, Australia; ^3^ Department of Pharmacy, Affiliated Cancer Hospital of Zhengzhou University/Henan Cancer Hospital, Zhengzhou 450003, P.R. China

**Keywords:** oral squamous cell carcinoma stem-like cells, SCC-9 cell line, microRNA-542-3p, integrin-linked kinase, TGFβ1/Smads signaling pathway

## Abstract

In this study, we investigated the effects of microRNA-542-3p (miR-542-3p) on ILK/TGF-β1/Smad2/3 signaling and oral squamous cell carcinoma (OSCC) progression. Levels of miR-542-3p were lower in OSCC tissues (n=108) than adjacent normal tissues, whereas levels of ILK, TGF-β1 and Smad2/3 were higher. Patients with undifferentiated tumors, advanced TNM stage and lymph node metastasis showed low miR-542-3p levels. This was accompanied by high ILK expression and poor survival. Dual luciferase reporter assays of SCC-9 cells showed that miR-542-3p inhibited *ILK* gene expression by binding to its 3’UTR at 233-240 bp. SCC-9 cells transfected with miR-542-3p mimics exhibited elevated miR-542-3p and decreased ILK, TGF-β1 and Smad2/3 expression. They also showed reduced self-renewal (fewer CD44^+^ cells and tumor-spheres), invasiveness, migration, proliferation and survival. Conversely, miR-542-3p inhibitors promoted increased self-renewal (more CD44^+^ cells and tumor-spheres), invasiveness, migration, proliferation and survival. In xenograft experiments with nude mice, SCC-9 cells transfected with miR-542-3p mimics or siRNA-ILK yielded tumors with smaller volumes and weights than control tumors. These results demonstrate that miR-542-3p is a tumor suppressor that inhibits ILK/TGF-β1/Smad2/3 signaling, thereby inhibiting OSCC progression.

## INTRODUCTION

Oral cancer ranks sixth among all cancers with 90% of oral cancer patients diagnosed as oral squamous cell carcinoma (OSCC) [1]. It includes malignancies in the oral cavity, lip and pharynx. OSCC has the highest mortality rates among all carcinomas and is the most common head and neck cancer [1, 2]. The incidence of OSCC is between the ages of 45 and 75 years, and is gradually increasing [3, 4]. The etiology of OSCC involves both intrinsic and extrinsic factors with smoking, alcohol consumption and human papilloma virus infection being the main risk factors [5]. Poor therapeutic response, recurrence and metastasis are commonly encountered despite considerable advances in surgery, radiotherapy and chemotherapy [6]. OSCC progression involves multistep transformational changes with multiple genetic mutations [7]. In recent years, many biomarkers have been investigated to improve the power and cost-effectiveness of clinical applications. These include miRNAs that have been recognized as novel targets in OSCC diagnosis and therapy [8].

MicroRNAs (miRNAs) are short (17∼25 nucleotides) non-coding RNAs that regulate gene expression through the posttranscriptional repression of their target mRNAs and influence various physiological and pathological processes [9-11]. They regulate cell proliferation, differentiation, apoptosis, angiogenesis, stress resistance and self-renewal of stem cells [12]. The microRNA-542-3p (miR-542-3p) has been recognized as a tumor suppressor gene in numerous cancers [13, 14]. Transforming growth factor-β1 (TGF-β1) plays an important part in human diseases by downstream activation of TGF-β1/Smad signaling pathway and is secreted by many cell types [11]. TGF-β1/Smad signaling pathway is a major signaling pathway that regulates cancer cell growth and proliferation [15]. Integrin-linked kinase (ILK) regulates many key biological processes including cell cycle, growth and angiogenesis; its high expression enhances tumorigenesis [16-18]. Over expression of ILK is associated with the recurrence and poor survival for OSCC patients [19]. ILK is also the target gene of miR-542-3p [20]. A previous study demonstrated that miR-204-5p regulated proliferation and metastasis of OSCC cells by inhibiting CXCR4 [21]. MiR-483-5p was considered as an independent prognostic factor, and its high expression in OSCC patients had diagnostic and prognostic significance for OSCC [22]. Although miR-542-3p serves as a tumor suppressor in esophageal squamous cell carcinoma (ESCC), its role in OSCC is unclear [23]. Therefore, in this study, we investigated the significance of miR-542-3p in OSCC progression and survival through ILK/TGF-β1/Smad2/3 signaling pathway.

## RESULTS

### Expression of miR-542-3p, ILK, TGF-β1 and Smad2/3 proteins in OSCC tissues

MiR-542-3p expression was decreased in OSCC tissues (0.67 ± 0.14) compared to adjacent normal tissues (0.91 ± 0.05; *P* < 0.05; Figure 1A). Conversely, OSCC tissues had increased ILK mRNA levels (1.76 ± 0.39) compared to adjacent normal tissues (0.94 ± 0.19; *P* < 0.05; Figure 1A). Western blotting analysis showed increased ILK, TGF-β1 and Smad2/3 protein expression in OSCC tissues compared to adjacent tissues (all *P* < 0.05; Figure 1B). Immunohistochemical analysis demonstrated cytoplasmic and diffuse distribution of ILK protein; its expression was higher in OSCC tissues compared to adjacent normal tissues (*P* < 0.05; Figure 1C-1D).

**Figure 1:** MiR-542-3p, ILK, TGF-β1 and Smad2/3 expression in OSCC tissues **(A)** RT-PCR analysis of miR-542-3p and ILK mRNA levels in OSCC and adjacent normal tissues is shown. **(B)** Western blot analysis of ILK, TGF-β1, and Smad2/3 proteins in OSCC and adjacent normal tissues is shown. **(C)** Representative images (40X) showing immunohistochemical staining of ILK in OSCC and adjacent normal tissues are shown. **(D)** Quantitative analysis of ILK protein expression in OSCC tissue samples (n = 108, each sample repeated thrice) is shown. Note: * denotes *P* < 0.05 compared with adjacent normal tissues. miR-542-3p, microRNA-542-3p; ILK, integrin-linked kinase; OSCC, oral squamous cell carcinoma; qRT-PCR, quantitative real-time polymerase chain reaction; TGF-β1, transforming growth factor-beta-1; GAPDH, glyceraldehyde-3-phosphate dehydrogenase.

### Correlation between miR-542-3p, ILK and clinicopathological features of OSCC patients

As shown in Table 1, miR-542-3p expression correlated with the TNM stage (both *P* < 0.05), but not with gender, age, history of smoking, tumor size or histological differentiation in OSCC patients (all *P* > 0.05). ILK protein expression correlated with the histological differentiation, TNM stage and lymph node metastasis (all *P* < 0.05), but not with gender, age, history of smoking or tumor size (all *P* > 0.05).

**Table 1:** Associations of miR-542-3p and ILK protein expressions with the clinicopathological features of patients with OSCC

Clinicopathological features	Case	miR-542-3p (relative expression)	*P*	ILK (positive rate)	*P*
Age (years)					
< 60	42	0.69 ± 0.14	0.471	33.42 ± 18.26	0.706
≥ 60	66	0.67 ± 0.14		32.06 ± 18.21	
Gender					
Male	79	0.66 ± 0.13	0.092	33.22 ± 18.30	0.554
Female	29	0.71 ± 0.15		30.87 ± 17.98	
Tumor size					
< 3 cm	47	0.66 ± 0.15	0.305	31.98 ± 18.07	0.761
≥ 3 cm	61	0.69 ± 0.15		33.06 ± 18.36	
History of smoking					
Yes	69	0.69 ± 0.14	0.157	32.57 ± 18.65	0.994
No	39	0.65 ± 0.14		32.60 ± 18.01	
Differentiation					
Moderately or highly differentiated	64	0.74 ± 0.11	< 0.001	28.23 ± 17.49	0.002
Poorly differentiated or undifferentiated	44	0.58 ± 0.11		38.94 ± 17.40	
Lymph node metastasis					
Yes	59	0.75 ± 0.10	< 0.001	27.94 ± 17.52	0.003
No	49	0.58 ± 0.11		38.19 ± 17.47	
TNM Stage					
I/II Stage	60	0.75 ± 0.10	< 0.001	28.36 ± 17.66	0.006
III/IV Stage	48	0.58 ± 0.11		37.88 ± 17.55	

Note: MiR-542-3p, microRNA-542-3p; ILK, integrin-linked kinase; OSCC, oral squamous cell carcinoma; TNM, tumor-node-metastasis.

### Association between miR-542-3p and ILK, TGF-β1 and Smad2/3 proteins

Spearman correlation analysis showed that miR-542-3p levels negatively correlated with ILK (r = -0.351, *P* < 0.001), TGF-β1 (r = -0.658, *P* <0.001) and Smad2/3 (r = -0.247, *P* = 0.010) expression (Figure 2A-2C).

**Figure 2:** Association between miR-542-3p and ILK, TGF-β1 and Smad 2/3 expression in OSCC tissues Correlation analysis between miR-542-3p and **(A)** ILK **(B)** TGF-β1 and **(C)** Smad 2/3 protein levels in OSCC patient tissues (n=108) is shown. miR-542-3p, microRNA-542-3p; ILK, integrin-linked kinase; OSCC, oral squamous cell carcinoma; TGF-β1, transforming growth factor-beta-1.

### Risk factors for prognosis of OSCC patients

Kaplan-Meier survival curves showed that patients with low miR-542-3p expression (average expression of miR-542-3P was 0.67, which used as cutoff value) had lower survival rates compared to high miR-542-3p expression group (Figure 3A). Similarly, patients with high ILK expression (20% used as cutoff value) had lower survival compared to those with low ILK expression (Figure 3B). Kaplan-Meier survival curves based on clinicopathological factors showed that (1) patients in III/IV stages had lower survival compared to those in the I/II stages; (2) patients with low differentiation tumors had lower survival rates compared to those with the moderate and high differentiation tumors; and (3) patients with lymph node metastasis had lower survival rates compared to those without lymph node metastasis (Figure 3C-3E). COX proportional hazard model analysis showed that miR-542-3p and ILK expression and lymph node metastasis indicated poor prognosis for OSCC patients (both *P* < 0.05; Table 2).

**Figure 3:** Kaplan-Meier survival curve analysis of OSCC risk factors Kaplan-Meier curves showing survival characteristics based on **(A)** high and low miR-542-3p expression, **(B)** high and low ILK protein expression, **(C)** early and advanced TNM stages and **(D)** degree of differentiation (undifferentiated versus moderate or highly differentiated) in OSCC patient tissues and **(E)** presence or absence of lymph node metastasis is shown.

**Table 2:** Results of multivariate COX regression analysis of patients with OSCC

Factors	*B*	*SE*	*Wald*	*EXP*	*P*	95% *CI*	
						Lower	Upper
miR-542-3p	1.777	0.54	10.842	5.913	0.001	2.053	17.03
ILK	1.763	0.642	7.548	5.831	0.006	1.658	20.515
TNM stage	-0.264	0.451	0.342	0.768	0.559	0.317	1.861
Differentiation	-1.431	1.281	1.248	0.239	0.264	0.019	2.945
lymphatic metastasis	2.692	1.106	5.922	14.768	0.015	1.689	129.166

Note: MiR-542-3p, microRNA-542-3p; COX, Cox’s proportional hazards regression model; ILK, integrin-linked kinase; 95%CI, 95% confidence interval; TNM, tumor-node-metastasis; SE, standard error.

### MiR-542-3p binds to 3’UTR of *ILK*

The miR-542-3p binding site in *ILK* gene was located in the 3’UTR by the Target Scan software (Figure 4A). The mutant and wild-type sequences of *ILK*-3’UTR were designed and inserted a luciferase reporter plasmid into them. SCC-9 cells co-transfected with miR-542-3p mimics and mutant (Mut-miR-542-3p/ILK) recombinant plasmid showed no significant effect on luciferase activity (*P* > 0.05), whereas luciferase activity decreased in SCC-9 cells with Wt-miR-542-3p/ILK plasmid (*P* < 0.05) indicating that miR-542-3p negatively regulated ILK (Figure 4B).

**Figure 4:** Dual luciferase reporter analysis of miR-542-3p binding to 3’UTR of *ILK* gene **(A)** Target Scan prediction of miR-542-3p binding site in 3’UTR of *ILK* gene. **(B)** Dual luciferase reporter gene assay showing miR-542-3p activity in presence of *ILK* gene with wild type or mutant miR-542-3p binding site is shown. Note: * denotes *P* < 0.05 compared with the blank group; each experiment was repeated thrice.

### MiR-542-3p inhibits CD44^+^SCC-9 cell growth and self-renewal

Compared to the blank (71.37%) and mimic control (69.86%) groups, CD44^+^ SCC-9 cells decreased in the miR-542-3p mimics (31.21%) and siRNA-ILK (42.37%) groups (all *P* < 0.05). This showed that the overexpression of miR-542-3p inhibited SCC-9 cell growth. In comparison, there was increased proportion of CD44^+^ SCC-9 cells in the miR-542-3p inhibitors group (93.12%; all *P* < 0.05; Figure 5A). Tumor-sphere formation assay demonstrated self renewal ability of SCC-9 cells. Compared with the blank group (31.04% ± 0.86%), there were lower number of tumor spheres in the miR-542-3p mimics (19.86% ± 0.61%) and siRNA-ILK (21.18% ± 0.86%) groups, and increased number of tumor spheres in the miR-542-3p inhibitors group (51.31% ± 2.13%; all *P* < 0.05; Figure 5B). Moreover, compared to the miR-542-3p inhibitors group, the number of tumor spheres decreased in the miR-542-3p inhibitors + siRNA-ILK group (40.37% ± 1.34%; *P* < 0.05). The numbers of tumor-spheres in the blank, mimic control and inhibitor control groups were similar (both *P* > 0.05).

**Figure 5:** Effects of differential miR-542-3p expression on SCC-9 cell proliferation and tumor sphere formation **(A)** Numbers of CD44^+^ SCC-9 cells in (1) blank (2) miR-542-3p mimics (3) mimics control (4) miR-542-3p inhibitors (5) inhibitors control (6) small interfering RNA (siRNA)-ILK and (7) miR-542-3p inhibitors + siRNA-ILK groups, 48h after transfection. **(B)** Total number of tumor spheres in (1) blank (2) miR-542-3p mimics (3) mimics control (4) miR-542-3p inhibitors (5) inhibitors control (6) small interfering RNA (siRNA)-ILK and (7) miR-542-3p inhibitors + siRNA-ILK SCC-9 cell groups. Note: Each experiment was repeated thrice; * denotes *P* < 0.05 compared with the blank group.

### Expression of miR-542-3p, ILK, TGF-β1 and Smad2/3 in SCC-9 cells

We observed that expression of miR-542-3p, ILK and TGF-β1/Smad signaling pathway-related proteins was similar in mimic control, inhibitor control, si-ILK and the blank groups (all *P* > 0.05; Figure 6). Compared with the blank group, miR-542-3p levels increased in the miR-542-3p mimics group and decreased in the miR-542 inhibitors and the miR-542-3p inhibitors + si-ILK groups (both *P* < 0.05; Figure 6A). Compared with the mimic group, ILK mRNA and protein levels as well as TGF-β1 and Smad2/3 protein levels decreased in the miR-542-3p and si-ILK groups and increased in the miR-542-3p inhibitors group (all *P* < 0.05; Figure 6A-6C). Moreover, ILK, TGF-β1and Smad2/3 protein levels in the miR-542-3p + siRNA-ILK group were between miR-542-3p inhibitors and blank group levels (all *P* < 0.05; Figure 6B-6C). Therefore, these data indicated that miR-542-3p inhibited ILK protein expression, which correlated with the expression of TGF-β1 and Smad2/3 proteins. Hence, miR-542-3p inhibited ILK/TGF-β1/Smad signaling pathway.

**Figure 6:** Effects of differential miR-542-3p expression on ILK, TGF-β1 and Smad2/3 protein expression **(A)** Expression of miR-542-3p and ILK mRNA in (1) blank (2) miR-542-3p mimics (3) mimics control (4) miR-542-3p inhibitors (5) inhibitors control (6) small interfering RNA (siRNA)-ILK and (7) miR-542-3p inhibitors + siRNA-ILK groups. **(B)** Representative western blots showing ILK, TGF-G1 and Smad2/3 protein levels in SCC-9 cell groups 1-7. **(C)** Quantitative analysis of ILK, TGF-G1 and Smad2/3 protein levels in SCC-9 cell groups 1-7. Note: Each experiment was repeated thrice; * denotes *P* < 0.05 compared with the blank group; # denotes *P* < 0.05 compared with the miR-542-3p inhibitors group.

### MiR-542-3p decreases SCC-9 cell proliferation

MTT assay demonstrated that cell proliferation was similar in the mimic control, inhibitor control, si-ILK and the blank groups (*P* > 0.05; Figure 7). Moreover, cell proliferation decreased in the miR-542-3p mimics and si-ILK groups and increased in the miR-542-3p inhibitors group (*P* < 0.05; Figure 7). In the miR-542-3p inhibitors + si-ILK group, cell proliferation was between the blank and the miR-542-3p inhibitors groups (*P* < 0.05; Figure 7). These data indicated that miR-542-3p inhibition of ILK expression decreased SCC-9 cell proliferation.

**Figure 7:** Effects of differential miR-542-3p expression on SCC-9 cell proliferation Analysis of SCC-9 proliferation by MTT assay in (1) blank (2) miR-542-3p mimics (3) mimics control (4) miR-542-3p inhibitors (5) inhibitors control (6) small interfering RNA (siRNA)-ILK and (7) miR-542-3p inhibitors + siRNA-ILK groups. Note: Each experiment was repeated thrice; * denotes *P* < 0.05 compared with the blank group; # denotes *P* < 0.05 compared with the miR-542-3p inhibitors group.

### MiR-542-3p inhibits SCC-9 cell migration

Compared with the blank group (0.78 ± 0.07), SCC-9 cell migration decreased in the miR-542-3p mimics (0.35 ± 0.10) and siRNA-ILK (0.44 ± 0.11) groups and increased in the miR-542-3p inhibitors group (1.41 ± 0.12; all *P* < 0.05; Figure 8A-8B). There was no significant difference in cell migration between the mimic control, the inhibitor control and the blank groups (both *P* > 0.05). The cell migration level in the inhibitors + siRNA-ILK group was between the miR-542-3p inhibitors and the blank groups (both *P* < 0.05). These data indicated that overexpression of miR-542-3p inhibited SCC-9 cell migration.

**Figure 8:** Effects of differential miR-542-3p expression on SCC-9 cell migration **(A)** Scratch test analysis of SCC-9 cell migration in (1) blank (2) miR-542-3p mimics (3) mimics control (4) miR-542-3p inhibitors (5) inhibitors control (6) small interfering RNA (siRNA)-ILK and (7) miR-542-3p inhibitors + siRNA-ILK groups. **(B)** Quantification of the width of scratch in groups 1-7. Note: All experiments were repeated thrice; * denotes *P* < 0.05 compared with the blank group; # denotes *P* < 0.05 compared with the miR-542-3p inhibitors group.

### MiR-542-3p reduces SCC-9 cell invasiveness

Transwell migration assay showed that the number of invading cells in the blank (116.31 ± 11.12) the mimic control (121.68 ± 14.41) and inhibitor control (122.76 ± 9.24) groups were similar (both *P* > 0.05). However, the SCC-9 cell invasiveness decreased in the miR-542-3p mimics (59.38 ± 7.55) and siRNA-ILK (71.13 ± 6.52) groups, but increased in the miR-542-3p inhibitors (198.63 ± 17.62) group (all *P* < 0.05; Figure 9A-9B). The number of invading cells in the miR-542-3p inhibitors + siRNA-ILK group (163.37 ± 13.19) was between the miR-542-3p inhibitors and the blank groups (both *P* < 0.05; Figure 9A-9B).

**Figure 9:** Effects of differential miR-542-3p expression on SCC-9 cell invasiveness **(A)** Representative images (200X) of Transwell assay showing invasion ability of SCC-9 cells from (1) blank (2) miR-542-3p mimics (3) mimics control (4) miR-542-3p inhibitors (5) inhibitors control (6) small interfering RNA (siRNA)-ILK and (7) miR-542-3p inhibitors + siRNA-ILK groups. **(B)** Quantitative analysis of total number of invading cells in SCC-9 cell groups 1-7. Note: All experiments were repeated thrice; * denotes *P* < 0.05 compared with the blank group; # denotes *P* < 0.05 compared with the miR-542-3p inhibitors group.

### MiR-542-3p reduces SCC-9 cell cycling and increases apoptosis

Cell cycle profiles were similar in the blank, mimics control and inhibitors control groups (all *P* > 0.05; Figure 10A-10B). Compared with the blank group, miR-542-3p mimics and the siRNA-ILK groups showed increased G0/G1 and decreased S and G2/M phase cells (all *P* < 0.05), whereas the miR-542-3p inhibitors group showed decreased G0/G1 and increased S and G2/M phase cells (all *P* < 0.05; Figure 10A-10B). Cell cycle distribution in the miR-542-3p inhibitors + si-ILK group was between the blank and the miR-542-3p inhibitor groups (*P* < 0.05; Figure 10A-10B). These results suggested that miR-542-3p inhibition increased SCC-9 cell cycling, whereas its upregulation resulted in G0/G1 cell cycle arrest.

**Figure 10:** Effects of differential miR-542-3p expression on SCC-9 cell cycle and apoptosis **(A)** Representative plots of SCC-9 cell cycle in (1) blank (2) miR-542-3p mimics (3) mimics control (4) miR-542-3p inhibitors (5) inhibitors control (6) small interfering RNA (siRNA)-ILK and (7) miR-542-3p inhibitors + siRNA-ILK groups. **(B)** Representative FACS plots showing percent (%) apoptosis of SCC-9 cells in groups 1-7. **(C)** Analysis of percent G0/G1, S and G2/M phase cells of SCC-9 cells in groups 1-7. **(D)** Analysis of percent apoptosis of SCC-9 cells in groups 1-7. Note: All experiments were repeated thrice; * denotes *P* < 0.05 compared with the blank group; # denotes *P* < 0.05 compared with the miR-542-3p inhibitors group.

Flow cytometry analysis of apoptosis showed no differences in the blank (14.76 % ± 0.76%), mimics control (14.65% ± 0.81%) and the inhibitors control (15.22 %± 0.86%) groups (*P* > 0.05; Figure 10C-10D). However, apoptosis increased in the miR-542-3p mimics (25.19% ± 0.79 %) and the si-ILK (25.36% ± 1.53%) groups and decreased in the miR-542-3p inhibitors (5.43% ± 0.86%) group (*P* < 0.05; Figure 10C-10D). Apoptosis rate in the miR-542-3p inhibitors + si-ILK group (10.14% ± 0.97%) was between the blank and the miR-542-3p inhibitors groups (both *P* < 0.05; Figure 10C-10D).

### MiR-542-3p mimics and ILK siRNA inhibit SCC-9 xenograft tumor growth in nude mice

As shown in Figure 11A-11B, the tumor volume and weight in nude mice xenografted with SCC-9 cells transfected with miR-542-3p mimics and siRNA-ILK groups were similar (*P* > 0.05) and lower compared to the control group (all *P* < 0.05).

**Figure 11:** Effects of differential miR-542-3p and ILK expression on xenograft tumor growth in nude mice **(A)** Total tumor volume of xenografted control, miR-542-3p mimic and siRNA-ILK transfected SCC-9 cells in nude mice. **(B)** Representative images of control, miR-542-3p mimic and siRNA-ILK SCC-9 cell tumors in nude mice. **(C)** Total weight of control, miR-542-3p mimic and siRNA-ILK SCC-9 cell tumors in nude mice. Note: * denotes *P* < 0.05 compared with the control group.

## DISCUSSION

In this study, we analyzed the role of miR-542-3p in OSCC progression. We demonstrated that miR-542-3p regulates TGF-β1/Smad2/3 signaling pathway by inhibiting ILK expression. We observed reduced miR-542-3p levels in OSCC tissues and increased ILK mRNA and protein levels along with elevated TGF-β1 and Smad2/3 protein levels compared to adjacent normal tissues. Moreover, overexpression of miR-542-3p inhibited the TGF-β1/Smad signaling pathway by down-regulating ILK and diminished self-renewal, differentiation, proliferation and survival of SCC-9 cells.

MiR-542-3p has a tumor suppressor role in osteoblast cells and ESCC tissues, and gastric and bladder cancers [13, 23-25]. Recent studies showed low miR-542-3p expression in bladder cancer tissues; its inhibition promoted tumor cell growth [13, 14]. Dual-luciferase reporter gene assay demonstrated that ILK was the target gene of miR-542-3p and overexpression of miR-542-3p negatively regulated ILK expression. Oneyama *et al.* also demonstrated that miR-542-3p performed tumor suppressor function in many human tumors and controlled ILK-mediated cell adhesion and invasion during tumor progression [20].

Most importantly, we demonstrated that miR-542-3p inhibition increased the proportion of CD44^+^ SCC-9 cells, which suggested that miR-542-3p inhibited the proliferation of SCC-9 cells. Besides, compared with the blank group, the numbers of tumor spheres decreased in the miR-542-3p mimics and siRNA-ILK groups and increased in the miR-542-3p inhibitors group. Moreover, compared with the miR-542-3p inhibitors group, the number of tumor spheres decreased in the miR-542-3p inhibitors + siRNA-ILK group. This suggested that miR-542-3p inhibited self-renewal and differentiation of SCC-9 cells by down-regulating ILK/TGF-β1/Smad2/3 signaling pathway. Tumor sphere expands and enriches tumor cells, and tumor sphere formation is analyzed to test self-renewal and differentiation of stem cells [26].

Cancer stem cells (CSCs) are either derived from transformation of normal stem cells that possess self-renewal capacity or from differentiated cells that acquire self-renewal properties as a result of genetic or epigenetic alterations [27]. The CSCs share characteristics of normal stem cells including self-renewal, ability to differentiate and activate anti-apoptotic pathways. Hence, CSCs can initiate tumors that are resistant to chemotherapy and metastasize to other tissues where they further differentiate and generate tumors [28]. The overexpression of miR-542-3p significantly inhibited the activation of β-catenin and nuclear factor-κB signaling pathways that promote carcinogenesis [25]. TGF-β signaling pathway also plays a very critical role in regulating cell growth, differentiation, and development of biological systems [29, 30]. TGF-β1 promotes tumor cell growth through the Smad-ILK signaling pathway by increasing Smad2/3 and ILK expression [31]. TGF-β1 expression is regulated by ILK activation, which responds to various pathological and physiological stimuli via TGF-β1 [32].

Additionally, our study found that miR-542-3p inhibited the SCC-9 cell proliferation by suppressing ILK expression. Inhibition of ILK resulted in treatment-related delays in tumor growth, reduced tumor angiogenesis and functionality of tumor vasculature [33]. Moreover, overexpression of miR-542-3p inhibited the migration and invasion of SCC-9 and arrested SCC-9 cells in G0/G1 phase. Also, overexpression of miR-542-3p and low expression of ILK promoted apoptosis of SCC-9 cells. A previous study showed that miR-542-3p expression decreased cell proliferation by inhibiting G1 and G2/M cell cycle phases [34]. MiR-542-3p was a tumor suppressor in melanomas by reducing cell migration and invasion [35]. Our study showed decreased invasion of SCC-9 cells in the miR-542-3p mimics and siRNA-ILK groups. This suggested that over expression of miR-542-3p and low expression of ILK decreased the invasion of SCC-9 cells. ILK regulates cell proliferation, differentiation, migration and apoptosis [36]. ILK plays critical roles in progression and metastasis of OSCC, and is a critical prognostic indicator for OSCC patients [36]. Bedal *et al.* demonstrated that high expression of ILK promoted tumor invasion, tumor grade, clinical stage and positive lymph node status, and increased the risk and complications of disease recurrence in OSCC [37]. The over expression of ILK improved the invasiveness of tumor cells by inducing the expression of invasion-related genes [38, 39]. Since our study was based on only one cell line, namely, SCC-9, further clinical research is necessary to demonstrate the efficacy of treating OSCC by regulating miR-542-3p. Also, the role of TGF-β1/Smad signaling pathway on the proliferation and survival of OSCC cells needs further experimentation.

In conclusion, our study demonstrates that overexpression of miR-542-3p inhibits TGF-β1/Smad2/3 signaling pathway by downregulating ILK. Therefore, miR-542-3p is a potential therapeutic target for OSCC.

## MATERIALS AND METHODS

### OSCC patient specimen

OSCC tissues were obtained from 108 patients who underwent surgical treatment in First Affiliated Hospital of Zhengzhou University and Henan Cancer Hospital/Affiliated Cancer Hospital of Zhengzhou University between August 2012 and December 2015. Among the 108 OSCC patients, 64 had moderately or highly differentiated squamous carcinoma and 44 were poorly differentiated or undifferentiated. The patients included 29 females and 79 males with an average age of 58.52 ± 14.47 years. Sixty-nine patients had a history of smoking and 49 patients had lymph node metastasis. Based on Tumor Node Metastasis (TNM) staging system of Union International Against Cancer (UIAC) in 2002, 60 cases were stage I/II and 48 were stage III/IV [40]. The normal tissues adjacent to the tumors were used as controls. The patients never had any radiotherapy, chemotherapy or related treatment before surgical treatment with complete clinical data. This study was approved by the Ethics Committee of First Affiliated Hospital of Zhengzhou University and Henan Cancer Hospital/Affiliated Cancer Hospital of Zhengzhou University. Informed consent was obtained from all study subjects and/or their legal guardians.

### Immunohistochemistry

The PV-9000 two-step method for immunohistochemical staining was used to determine the expression of ILK, TGF-β1 and Smad2/3 proteins in OSCC tissues. Each tissue microarray paraffin block was cut into serial 4μm sections, dewaxed and hydrated with gradient alcohol followed by antigen retrieval in a microwave. Endogenous peroxidase (PO) was blocked by incubation with 3% hydrogen peroxide (H_2_O_2_). Then, the sections were incubated with mouse anti-human ILK antibody (1:50; Wuhan Boster Biological Technology Ltd., Wuhan, China) at 4°C overnight. Then, they were incubated with polymerase auxiliary agent for 20 min at room temperature followed by horseradish peroxidase-labeled goat anti-mouse secondary antibody (Abcam, Cambridge, MA, USA) for 30 min at room temperature. Diaminobenzidine (DAB) (Sigma-Aldrich Biological Technology Co., Ltd., USA) was used for developing. The sections were counterstained with hematoxylin and sealed. Phosphate buffered saline (PBS) replaced the primary antibody in the negative control. The cells with visible yellow or brown cytoplasm or cell membrane were identified as positive. Four high power fields (× 400) were randomly selected in each slide and 200 OSCC cells were counted in each field. Proportion of positive cells was used to determine the scores. Cells with more than 25% brown and brownish yellow granules in the cytoplasm were designated as positive., Positive expression rate was defined as positive cell numbers relative to total cell numbers. The scoring was performed independently by two individuals who were blinded to the source of the specimens.

### Patient follow-up and overall survival

Follow-up was conducted by out-patient consultation or over the phone. The deadline of follow up was January 2017. Overall survival (OS) was defined as the time from first diagnosis to either death or the final time of follow-up (January 2017). At the end of follow-up (12 months), 101 patients completed follow-up data, whereas 7 patients died. Hence, the effective follow-up rate was 93.5.0%.

### SCC-9 cell culture

The SCC-9 cells (CRL-1629) (American Type Culture Collection [ATCC], VA, USA) were grown in Dulbecco’s modified Eagle medium (DMEM)/F12 medium (Gibco, Grand Island, NY, USA) with 10% fetal bovine serum (FBS). When the cell density reached 80-90%, the cells were digested by trypsin (Gibco, Grand Island, NY, USA) for single cell suspension. The cells were then centrifuged at 1500 rpm for 10 mins, and washed twice with PBS, and resuspended in 200μL PBS. Next, the cells were incubated with 100μl mouse anti-human CD44^+^ antibody (Cell Signaling Technologies (CST), Beverly, MA, USA) for 45 min. The cells were washed twice by PBS and resuspended in 200μL PBS. The SCC-9 cells were separated by flow cytometry (FACSCanto II) (BD Biosciences Company, NJ, USA) based on CD44 immunofluorescent labeling. The CD44^+^ cells corresponded to OSCC cells whereas the rest were non-stem-like cells. These cells were preserved and frozen for further use or used for further experiments.

### Dual-luciferase reporter gene assay

The putative miR-542-3p binding site in the *ILK* gene was identified at 233-240 bases of its 3’UTR by Target Scan (http://www.targetscan.org/vert_71). To confirm miR-542-3p binding to the 3’UTR site in ILK gene, genomic DNA was extracted from SCC-9 cell line according to the instructions of TIANamp Genomic DNA Kit (TIANGEN Biotechnology Co., Ltd, Beijing, China). We designed two 72bp sequences, (1) ILK-3’-UTR-wt with wild type miR-542-3p binding site (5’- CUCAGAGCUUUGUCACUUGCCACAUGGUGUCUCCCAACAUGGGAGGGAUCAGCCCCGCCUGUCACAAUAAAG-3’) and (2) ILK-3’-UTR-mut with mutated miR542-3p binding site (UCGAGCUUGGUUGUGACACAAUGGUUGGCCGCCACUUCUCACCAGCACAAACCGUCCUUGGGGACCGAGAGCU). Both ILK-3’-UTR-wt and ILK-3’-UTR-mut sequences were cloned into pMir-GLO vector with luciferase reporters and SCC-9 cells was transfected, after which detected with luciferase double reporter gene assay reagent (Promega Corporation, Madison, WI, USA).

The dual-luciferase reporter assay was performed to test the luciferase activity of samples. The primary medium was removed 48h after transfection. The SCC-9 cells were washed twice by PBS and lysed with 100 μl passive lysis buffer (PLB) at room temperature for 15 min. Then, the cell lysate was obtained. LARII and Stop & Glo® Reagent (100 μl) was added into the luminous tube or plate with 20μl cell lysate and the firefly and renilla luciferase activities were measured in a luminescence detector (Turner BioSystems Co, Ltd, USA, Model: Modulus™). The relative activity of the two luciferases was calculated (ΔCT). The experiment was repeated thrice.

### Transfection and cell grouping

The miR-542-3p mimics, miR-542-3p inhibitors, their corresponding controls and ILK siRNA (Shanghai Sangon Biotech Co. Ltd, China) were cloned into pEGFP-N1 vector. They were then transfected into the corresponding SCC-9 cells, thereby generating (1) blank (2) miR-542-3p mimics (3) mimics control (4) miR-542-3p inhibitors (5) inhibitors control (6) small interfering RNA (siRNA)-ILK and (7) miR-542-3p inhibitors + siRNA-ILK groups. The transfection protocol is shown in Table 3.

**Table 3:** Sequence for transfection

Gene	Sequence (5’-3’)
MiR-542-3p mimics	TGTGACAGATTGATAACTGAAA
Mimics control	UUCUCAGAAAGGUGAAAUUUAUU
MiR-542-3p inhibitors	TTTCAGTTATCAATCTGTCACA
Inhibitors control	UUGUACUACACAAAAGUACUG
SiRNA-ILK	GGACACATTCTGGAAGGGG

Note: MiR-542-3p, microRNA-542-3p; ILK, integrin-linked kinase.

SCC-9 cells were grown in a 25 cm^2^ culture flask until cell density reached 30-50% in complete medium. Then, the cells were mixed with 100μl serum-free culture medium in sterile EP tubes and incubated with 5μl lipofectamine 2000 (Invitrogen Biotech Co., Ltd., New York, USA) for 5 min at room temperature. Then, 1μg DNA was diluted in culture medium without serum. The diluted lipofectamine 2000 and DNA mixture was mixed well and incubated for 20 min at room temperature to form DNA-liposome complexes. The cells in the culture flask were washed with culture medium without serum. Serum-free DMEM (with no antibiotics) was added to the DNA-liposome complexes and mixed with the cells such that plasmid concentration was 50nM. The transfected cells were grown in an incubator with 5% CO_2_ at 37°C. After 6∼8 h, the liquid was replaced and complete medium was added for continuous culture. The SCC-9 stem-like cells labeled with CD44^+^ were sorted out by flow cytometry.

### Quantitative real-time polymerase chain reaction (qRT-PCR)

Total RNA was extracted from the OSCC and adjacent normal tissues and SCC-9 cells by Trizol method. The optical density (OD) values at 260 nm and 280 nm were recorded by the ND-1000 ultraviolet-visible spectrophotometer (Nanodrop Technologies Inc., Wilmington, USA). The quality of total RNA was measured and the RNA concentration was adjusted in samples by diluting with ultra pure water. Then, 1μg RNA was reverse transcribed by two-step method according to instructions in the reverse transcription kit (Fermentas Inc., Hanover, MD, USA). The first strand cDNA synthesis conditions were as follows: 70°C for 10 min, ice bath for 2 min, 42°C for 60 min, 70°C for 10 min. The first strand cDNA samples were stored at -80 °C for further use.

The qRT-PCR reaction was performed according to the instructions of reverse transcription kit (Fermentas Inc., Hanover, MD, USA) using TaqMan probes. The primer sequences for qRT-PCR are presented in Table 4. The reaction conditions were as follows: pre-denaturation at 95°C for 30 s, denaturation at 95°C for 10 s, annealing at 60°C for 20 s, and extension at 70°C for 10 s (40 cycles). The qRT-PCR was performed in Bio-Rad iQ5 (Bio-Rad, Inc., Hercules, CA, USA). U6 was used as internal reference of miR-542-3p [41], and GAPDH was used as the internal reference of other target genes. 2^-ΔΔCt^ was used to calculate the relative expression of the targeted genes. Each experiment was performed in triplicates.

**Table 4:** Primer sequences for qRT-PCR

Gene	Primer sequence (5’-3’)
MiR-542-3p	F: GCGGCTGTGACAGATTGATAAC
	R: GTGCAGGGTCCGAGGT
ILK	GCACTCAATAGCCGTAGTG
	CCTACTTGTCCTGCATCTTC
GAPDH	GGCACAGTCAAGGCTGAGAATG
	ATGGTGGTGAAGACGCCAGTA
U6	CTCGCTTCGGCAGCACA
	AACGCTTCACGAATTTGCGT

Note: qRT-PCR, quantitative real-time polymerase chain reaction; miR-542-3p, microRNA-542-3p; ILK, integrin-linked kinase; GAPDH, glyceraldehyde-3-phosphate dehydrogenase.

### Western blotting

Total protein lysates from the OSCC and adjacent normal tissues and SCC-9 cells from the 7 groups were prepared using the RIPA lysis buffer (Beyotime Biotechnology Co., Shanghai, China). Protein concentration was quantified by BCA protein assay kit (Thermo Fisher Scientific, San Jose, California, USA). Equal amounts of protein lysates (20 μl) were boiled with SDS-PAGE buffer for 5 min at 100°C and separated on a 10% SDS-PAGE gel. and transferred into the PVDF membrane at 48 V for 3.5 h. The PVDF membranes were blocked with 5% bovine serum albumin (BSA) for 2 h at room temperature and then washed by 1× Tris-buffered saline with Tween20 (TBST). Then, the membranes were probed with primary antibodies namely, mouse anti-human ILK (1: 2000), TGF-β1 (1: 1000), Smad2/3 (1: 1000) and β-actin (1: 1000) (Cell Signaling Technologies, Beverly, MA, USA) that were prepared with 5% BSA for 1 h at room temperature and rinsed in 1× TBST. Then, the blots were incubated with secondary goat anti-rabbit antibody (1: 4000; Cell Signaling Technologies, Beverly, MA, USA) for an hour at room temperature, rinsed with 1 × TBST and then developed with ECL reagent. The protein bands were quantified relative to β-actin to determine the relative expression of the target proteins.

### MTT assay

Transfected SCC9 cells were harvested by digesting with 0.25% trypsin when they reached 80% confluence. Then, the cells were seeded into a 96-well plate at 3 × 10^3^∼6 × 10^3^ cells per well in 200μl medium (6 wells per condition). Then, 20μl of 5mg/ml MTT solution (Sigma, USA) was added to each well and the cells were further cultured for 4 h. Then, after aspirating out the medium, 150μl Dimethyl sulfoxide (DMSO) (Sigma Company, USA) was added and the plate was gently shaken for 10 min. The OD value of the lysates was measured at 490 nm in the enzyme linked immunosorbent assay instrument at 24, 48 and 72 h, respectively. Cell viability was determined from the standard curve that was concurrently generated.

### Migration assay of SCC-9 cells

The bottom of the 6-well plate was marked with lines every 0.5∼1 cm followed by seeding 3 × 10^4^ transfected SCC-9 cells for culture overnight. When the cells reached 80∼90% confluence, the cells were scratched perpendicular to the line. The cells were further cultured for 48 h. Eight fields with scratches were randomly selected and analyzed for cell movement around the scratch in each well and photographed. Then the Motic Images Advanced 3.2 software was used to measure the relative width of scratch to determine the migration ability of cells. Each experiment was repeated thrice.

### Transwell invasion assay

The matrigel (Corning Glass Works, Corning, N.Y., USA) was dissolved overnight at 4°C and then diluted with serum-free DMEM medium (1: 3). Then, 30μl diluted matrigel was added to the upper chamber of each Transwell chamber (Corning Incorporated, US) and the bottom chamber. The cell suspension (3 × 10^4^) was added into Transwell upper chamber, and 0.5 ml DMEM with 10% FBS was added to the lower chamber. After 48 h of culturing, the numbers of cells in the bottom chamber were photographed under the inverted microscope. The mean number of cells was determined by selecting 5 fields per well for each group. The total number of cells in each group passing through the matrigel represented the ability of invasion for the particular group. All experiments were repeated thrice.

### Flow cytometry

After transfection for 48 h, the SCC9 cells were harvested and fixed in cold 75% ethanol (chilled at -20°C) at 4°C overnight. After centrifugation, the cells were washed by cold PBS twice to remove excess ethanol. RNAase was added to the cell suspension and incubated in a water bath without light for 30 min followed by 5μg/ml propidiom iodide (PI) for staining and mixed well. The cells were then subjected to flow cytometry and the proportion of cells in G0/G1, S and G2/M phase of the cell cycle were analyzed from the FACS plots. Each experiment was performed in triplicate.

Annexin V/PI double staining was used to detect cellular apoptosis. The SCC-9 cells after 48 h of transfection were harvested, adjusted to 1 × 10^6^/ml in 0.5 ml binding buffer and incubated for 15 mins at room temperature in the dark with 1.25μl AnnexinV-FITC (Nanjing Keygen Biotech. Co., Ltd., Jiangsu, China). Then the cells were pelleted by centrifugation at 1000 rpm for 5 min. The cells were then re-suspended with 0.5 ml chilled binding buffer, followed by addition of 10μl PI and then analyzed by flow cytometry (BD Biosciences Company, NJ, USA).

### Tumorsphere formation assay

After trypsinization, the SCC-9 cells were washed twice with PBS and once with serum-free DMEM medium. Then, 1000 cells were seeded into a culture flask and grown for a week. The cells were photographed every 3 days under a microscope. Finally, the number of tumorspheres and the number of cells in each tumor sphere were counted and compared.

### Tumor xenografts in nude mice

Fifteen specific pathogen free (SPF) nude mice (Hunan Silaike Jingda Experimental Animal Co., Ltd., Changsha, China) that weighed between 18∼25g and 5∼6 weeks of age were maintained in a SPF sterile laminar flow chamber with constant temperature (22°C-25°C) and humidity (55 ± 5%), sterile food, water, and bedding. The mice were divided into the control, miR-542-3p mimic and siRNA-ILK groups (5 mice in each group). Then, they were injected with 0.2 ml of corresponding cell suspensions (10^6^/ml) at the back with a hypodermic needle. The maximum diameter (a) and the maximum transverse diameter (b) of tumors were measured every three days. The volume (V = ab^2^/2) of tumors was calculated, and other parameters like the diet, shape and defecation of the nude mice was documented. After 28 days, all mice were sacrificed by cervical dislocation and the tumor was surgically removed, weighed and the final tumor volume was calculated.

### Statistical analysis

Data were analyzed using the SPSS 21.0 software (SPSS Inc., Chicago, IL, USA). The experimental data was represented as mean ± SD. Comparison between multiple groups was analyzed using variance analysis. The two pair comparison was tested with least significant difference (LSD)-*t* test. Enumeration data were displayed as frequency. Categorical data were compared by chi square test and ranked data were displayed by rank sum test. Correlation was analyzed by Spearman correlation analysis; survival time was measured by Kaplan-Meier curve; comparison among groups was analyzed by Log-rank test; multivariate analysis was performed using Cox regression model. *P* < 0.05 indicated statistical significance.
